# Socioeconomic Inequality in the Prevalence of Autism Spectrum Disorder: Evidence from a U.S. Cross-Sectional Study

**DOI:** 10.1371/journal.pone.0011551

**Published:** 2010-07-12

**Authors:** Maureen S. Durkin, Matthew J. Maenner, F. John Meaney, Susan E. Levy, Carolyn DiGuiseppi, Joyce S. Nicholas, Russell S. Kirby, Jennifer A. Pinto-Martin, Laura A. Schieve

**Affiliations:** 1 Department of Population Health Sciences, University of Wisconsin School of Medicine and Public Health, Madison, Wisconsin, United States of America; 2 Department of Pediatrics, University of Wisconsin School of Medicine and Public Health, Madison, Wisconsin, United States of America; 3 Waisman Center, University of Wisconsin-Madison, Madison, Wisconsin, United States of America; 4 Department of Pediatrics, University of Arizona Health Sciences Center, Tucson, Arizona, United States of America; 5 Department of Pediatrics, University of Pennsylvania, Philadelphia, Pennsylvania, United States of America; 6 Department of Epidemiology, Colorado School of Public Health, University of Colorado Denver, Aurora, Colorado, United States of America; 7 Division of Biostatistics and Epidemiology, Departments of Neurosciences and Medicine, Medical University of South Carolina, Charleston, South Carolina, United States of America; 8 Department of Community and Family Health, University of South Florida, Tampa, Florida, United States of America; 9 School of Nursing and School of Medicine, University of Pennsylvania, Philadelphia, Pennsylvania, United States of America; 10 National Center on Birth Defects and Developmental Disabilities, Centers for Disease Control and Prevention, Atlanta, Georgia, United States of America; University of Cape Town, South Africa

## Abstract

**Background:**

This study was designed to evaluate the hypothesis that the prevalence of autism spectrum disorder (ASD) among children in the United States is positively associated with socioeconomic status (SES).

**Methods:**

A cross-sectional study was implemented with data from the Autism and Developmental Disabilities Monitoring Network, a multiple source surveillance system that incorporates data from educational and health care sources to determine the number of 8-year-old children with ASD among defined populations. For the years 2002 and 2004, there were 3,680 children with ASD among a population of 557 689 8-year-old children. Area-level census SES indicators were used to compute ASD prevalence by SES tertiles of the population.

**Results:**

Prevalence increased with increasing SES in a dose-response manner, with prevalence ratios relative to medium SES of 0.70 (95% confidence interval [CI] 0.64, 0.76) for low SES, and of 1.25 (95% CI 1.16, 1.35) for high SES, (*P*<0.001). Significant SES gradients were observed for children with and without a pre-existing ASD diagnosis, and in analyses stratified by gender, race/ethnicity, and surveillance data source. The SES gradient was significantly stronger in children with a pre-existing diagnosis than in those meeting criteria for ASD but with no previous record of an ASD diagnosis (p<0.001), and was not present in children with co-occurring ASD and intellectual disability.

**Conclusions:**

The stronger SES gradient in ASD prevalence in children with versus without a pre-existing ASD diagnosis points to potential ascertainment or diagnostic bias and to the possibility of SES disparity in access to services for children with autism. Further research is needed to confirm and understand the sources of this disparity so that policy implications can be drawn. Consideration should also be given to the possibility that there may be causal mechanisms or confounding factors associated with both high SES and vulnerability to ASD.

## Introduction

Population indicators of socioeconomic status (SES), such as household wealth or income and parental education and occupation, are strongly correlated with the health and development of children [1]. For many chronic childhood disorders and for developmental disabilities overall, the association with SES often is found to be inverse, such that population prevalence decreases with increasing levels of SES [2], [3]. Documentation of this pattern, as well as exceptions to it, might provide clues to causal mechanisms underlying specific disorders or point to disparities in access to services, including early access to services that can stem the progression of mild conditions.

In the case of autism and autism spectrum disorder (ASD), evidence for an association with SES has been mixed and more often in the opposite direction of that for other childhood disorders. In the earliest clinical descriptions of children with autism, Kanner noted a preponderance of “highly intelligent parents” [4]. A number of clinical [5]–[9] and population-based [10]–[16] studies subsequently have reported positive associations between autism or ASD and SES indicators such as parental education, occupation, or income. In addition, ecological analyses of school enrollment data have found significant inverse associations between school district level proportions of children receiving special education under the autism disability category and SES indicators such as the proportion of students reported to be economically disadvantaged [17] and county median household income [18]. However, a nearly equivalent number of studies, both clinical [19]–[23] and epidemiological [24]–[28], have failed to find associations between SES and ASD, and one case-control study found lower educational attainment of mothers of children with autism compared to controls [29].

A compelling argument has been made that the positive associations between SES and ASD prevalence that have been observed likely are due either in part or entirely to ascertainment bias [22]–[24], [30], [31]. For example, it has been suggested that “more parents of high social class families [have] the necessary information and financial resources to find their way to the specialized facilities” [23] and “a knowledgeable and determined parent of an autistic child [is] more likely to obtain an informed diagnosis” [24]. To evaluate the role of biased ascertainment, Wing [24] called for population-based studies large enough to allow stratified analyses and evaluation of socioeconomic differences among subgroups.

In a previous analysis [16] of data from one site participating in the Autism and Developmental Disabilities Monitoring (ADDM) Network, we found a positive association between ASD prevalence and SES, and concluded that there was a need for larger studies to evaluate whether the SES gradient is found only among children with a pre-existing ASD diagnosis — a finding which would support the hypothesis that the SES gradient is a result of ascertainment bias. Alternatively, evidence of a similar SES gradient among children meeting diagnostic criteria for ASD who had not previously been diagnosed or classified as having an ASD would suggest that the ASD-SES association might not be entirely due to ascertainment bias.

We designed the present study to examine—among a large, diverse, population-based sample of 8-year-old children in the United States in which ASD case status was determined regardless of whether a child had a pre-existing ASD diagnosis—whether the prevalence of ASD is associated with SES and, if so, whether the association is consistent across subgroups defined by race/ethnicity, gender, phenotypic characteristics, diagnosis, and data sources.

## Methods

### Study Design and Data Sources

We implemented a population-based cross-sectional design in which data from 12 participating ADDM Network sites were analyzed [32]. The ADDM Network, established by the Centers for Disease Control and Prevention in 2000, is a population-based surveillance program operating in selected geographic locations in the United States. The surveillance program incorporates abstracted data from records of multiple educational and medical sources to determine the number of children who appear to meet the ASD case definition, regardless of pre-existing diagnosis. Clinicians determine whether the ASD case definition is met by reviewing a compiled record of all relevant abstracted data.

### Study Sample

Using the ADDM Network methodology, the network counted a total of 3680 8-year-old children as having an ASD in 2002 and 2004 in all study sites with available case and SES information, which were those located in Alabama, Arkansas, Arizona, Colorado, Georgia, Maryland, Missouri, North Carolina, New Jersey, Pennsylvania, South Carolina, and Wisconsin. ADDM Network data from the states of Utah and West Virginia were excluded because they did not include sufficient geographic indicators to allow SES classification.

The population denominator comprised 557 689 8-year-old boys and girls residing in the respective study areas in the two study years according to the 2000 U.S. Census [33]. We used the 2000 Census for both study years because it provided the most up-to-date socioeconomic information at the block group level. Compared with the 2000 Census, 2002 and 2004 intercensal estimates of population counts (which do not include relevant SES information at the block group level) were 3.9% lower. To estimate racial and racial/ethnic distributions, we multiplied the number of 8-year-olds within each census block group by the proportion of 6- to 11-year-olds in the same block group that were classified as non-Hispanic White, non-Hispanic Black or African American, Hispanic, Asian, or other. We then summed the block group frequencies of 8-year-old children in each racial/ethnic group. Compared with 8-year-old children nationally (as detailed in the 2000 U.S. Census), those in the study areas were more likely to be non-Hispanic Black or African American (28.6% vs. 15.7%) and less likely to be Hispanic (9.9% vs. 17.2%) (Table 1).

**Table 1:** Demographic Characteristics of ASD Cases, Population of 8-Year-Old Children in the Surveillance Area and Overall United States Population of 8-Year-Old Children.

		ASD Cases	Population of 8-Year-Old Children Residing in the Surveillance Area^a^	United States Population of 8-Year-Old Children^a^
Total		3680	557 689	4 179 230
% Male		81.4*	51.1	51.2
Race/Ethnicity	% Non-Hispanic White	60.1	57.8	60.3**
	% Non-Hispanic Black	24.6*	28.6	15.7**
	% Hispanic	7.7*	9.9	17.2**
	% Asian	2.6	2.3	3.3**
	% Other	1.7*	2.5	3.5**
	% Missing Race/Ethnicity	3.2*	0	0

a Based on 2000 Census data.

*p<0.05, comparing ASD cases to population of 8-year-old children residing in the surveillance area.

**p<0.05, comparing population of 8-year-old children residing in the surveillance area to United States population of 8-year-old children according to 2000 Census data.

### Case Definition

Autism spectrum disorder (ASD) refers to a group of neurodevelopmental disorders involving impairments in social interaction and communication, as well as the presence of repetitive or stereotyped behaviors. Specific disorders encompassed by ASD for which diagnostic criteria are provided by the Diagnostic and Statistical Manual Version IV-TR are autistic disorder, Asperger's disorder, and pervasive developmental disorder not otherwise specified [34]. Case status for the purpose of surveillance was determined based on a comprehensive review of educational and clinical records. Children were classified by experienced, trained clinician reviewers as having an ASD if they either had a documented previous classification of an ASD that was confirmed through review of diagnostic evaluation records or had an evaluation record from an educational or medical setting indicating behaviors consistent with Diagnostic and Statistical Manual Version IV-TR criteria for an ASD [34]. For children without a documented ASD classification, but with an indication of developmental delays or concerns consistent with a possible ASD classification, data were abstracted and systematically reviewed for all relevant ASD and developmental behaviors reported in the child's education or medical evaluations, or both, to determine whether behaviors described by qualified professionals in and across these evaluations were consistent with the Diagnostic and Statistical Manual Version IV-TR criteria.

Of the 3680 children with ASD, 2436 (66.2%) had a pre-existing ASD diagnosis. Of those with a pre-existing diagnosis, 1411 (58%) had a pre-existing diagnosis of autistic disorder, while information on the remaining 42% was insufficient to determine whether Diagnostic and Statistical Manual Version IV-TR criteria were met for autistic disorder versus pervasive developmental disorder not otherwise specified. Information from standardized intelligence tests was available for 75% of the children with ASD. Based on this information, children with an ASD were classified as having intellectual disability (IQ<70) versus normal range intelligence. Developmental regression was noted if the onset of ASD was characterized by loss of previously acquired skills in communication, social interaction or behavior. Further details regarding the ADDM Network methodology can be found in previous publications [32], [35].

### SES Indicators and Computation of SES-Specific Prevalence

To evaluate the association between SES and ASD, we implemented the following procedure to compute the prevalence of ASD in “Low SES,” “Medium SES,” and “High SES” tertiles of the population. We used three different approaches, each based on a different census indicator at the block group level, to identify population SES tertiles based on: (1) the percentage of families with children that had incomes above the federal poverty level (abbreviated here as “% above poverty”); (2) the percentage of adults 25 years of age or older who had a bachelor's degree (abbreviated here as “% bachelors”); and (3) median household income (“MHI”). The purpose of creating three sets of SES tertiles was to allow evaluation of consistency of the findings across different indicators.

To create the population SES tertiles, we: (1) weighted each census block group in the study areas by its number of 8-year-old residents; (2) ranked the census block groups by their values on the three census indicators (% above poverty, % bachelors, and MHI) and computed percentiles for each indicator; and (3) classified the block groups and thus the denominator of 8-year-olds into SES tertiles based on their percentiles. The result was three sets of population SES tertiles, one based on each indicator.

In the absence of current individual-level measures of SES in the ADDM Network surveillance database, we attached area-based SES measures to each child with ASD, using the approach described by Krieger and colleagues [36], based on census block group of residence of the child at the age of eight years. After geocoding each case, we classified the case into high SES, medium SES, or low SES categories based on the child's census block group values for the indicators % above poverty, % bachelors, and MHI. We then computed the SES-specific prevalence of ASD per 1 000 by dividing the number of children with ASD in each SES category by the general population in the same category.

### Statistical Analysis

To allow formal testing of a dose-response relationship between SES and ASD risk, we computed prevalence ratios with medium SES serving as the reference category, and Cochran-Armitage trend tests. We used SAS version 9.1 for all statistical analyses. We computed χ^2^ tests and 95% confidence intervals based on a Poisson distribution and log-link function [37]. To test for differences in SES between ASD cases and the surveillance population, we computed t-tests for the indicators % poverty and % bachelors, and the two-sample median test for the indicator MHI.

To evaluate whether the associations between SES and ASD varied by race/ethnicity, gender, phenotypic characteristics, pre-existing diagnosis of an ASD, and ascertainment sources of information, we performed stratified analyses and χ^2^ tests both of the SES gradient within strata and of the difference in the SES distribution of cases across strata, using the % above poverty indicator for SES. We chose this indicator for the stratified analyses after determining that the results were similar for all three SES indicators, and because the % above poverty block group indicator has been shown in previous studies to be correlated with a range of other measures of SES among the general population [36].

In addition to use of the indicator ‘*% above poverty’* in analyses presented in Tables 2 and 3, we have provided information in Table 1 about the ‘*percentage of the population residing in poverty areas*,’ where poverty areas are defined by the U.S. Census to include census block groups in which more than 20% of families with children have incomes below the poverty level [38].

**Table 2:** Socioeconomic Indicators for ASD Cases and the Population of 8-Year-Old Children in the Surveillance Area.

		ASD Cases	Population of 8-Year-Old Children Residing in the Surveillance Area^a^
Overall	% Living in a Poverty Area^b^	16.8*	25.8
	% of Adults with Bachelor's Degree	30.3*	24.8
	MHI (US$)	50 114*	42 898
Non-Hispanic White	% Living in a Poverty Area^b^	8.0*	10.5
	% of Adults with Bachelor's Degree	34.1*	29.8
	MHI (US$)	56 273*	51 890
Non-Hispanic Black	% Living in a Poverty Area^b^	36.1*	51.1
	% of Adults with Bachelor's Degree	21.5*	16.5
	MHI (US$)	38 833*	31 339
Hispanic	% Living in a Poverty Area^b^	31.7*	42.0
	% of Adults with Bachelor's Degree	21.2*	17.5
	MHI (US$)	40 910*	36 075
Asian	% Living in a Poverty Area^b^	8.3*	17.4
	% of Adults with Bachelor's Degree	42.2*	35.0
	MHI (US$)	59 892*	50 595

a Based on 2000 Census data.

b Poverty areas include census block groups in which more than 20% of families with children have incomes below the poverty level [36].

*p<0.05, comparing ASD cases to population of 8-year-old children residing in the surveillance area.

**Table 3:** Prevalence (95% CI^a^) of ASD per 1,000 8-Year-Olds and Ratios of ASD Prevalence by SES^b^, Stratified by Race/Ethnicity^c^.

		Non-Hispanic White	Non-Hispanic Black	Hispanic	Asian
Prevalence (95% CI)	Overall	6.9 (6.6, 7.3)	5.7 (5.3, 6.0)	5.1 (4.5, 5.7)	7.6 (6.1, 9.1)
	Low SES	5.7 (5.0, 6.4)	4.1 (3.7, 4.6)	4.0 (3.2, 4.8)	3.9 (1.6, 6.3)
	Medium SES	6.5 (6.0, 7.0)	6.8 (6.0, 7.6)	5.4 (4.3, 6.5)	6.0 (3.7, 8.3)
	High SES	7.7 (7.2, 8.1)	9.8 (8.4, 11.2)	7.5 (5.9, 9.2)	10.7 (7.9, 13.4)
	χ^2^ p-value	<0.0001	<0.0001	<0.0001	<0.0011
	trend test p-value	<0.0001	<0.0001	<0.0001	<0.0003
Prevalence Ratio (95% CI)	Low SES	0.88 (0.77, 1.02)	0.61 (0.52, 0.70)	0.74 (0.56, 0.97)	0.66 (0.33, 1.34)
	Medium SES	Reference	Reference	Reference	Reference
	High SES	1.18 (1.08, 1.30)	1.44 (1.21, 1.71)	1.40 (1.04, 1.89)	1.80 (1.13, 2.85)

a CI = confidence interval.

b Socioeconomic Status (SES) is indicated by the percentage of families with incomes above the federal poverty level who had children in the census block group of the index child, divided into population SES tertiles.

c The following differences in prevalence between ethnic group were statistically significant at p<0.05:

Overall: Non-Hispanic White versus Non-Hispanic Black; Non-Hispanic White versus Hispanic; Non-Hispanic Black versus Asian; and Hispanic versus Asian. In addition, the overall prevalence of ASD differs at p<0.05 across race/ethnic groups.

Low SES: Non-Hispanic White versus Non-Hispanic Black; Non-Hispanic White versus Hispanic; and Non_Hispanic White versus Asian. In addition, within the low SES stratum, the prevalence of ASD differs at p<0.05 across race/ethnic groups.

Medium SES: Non-Hispanic Black versus Hispanic.

High SES: Non-Hispanic White versus Non-Hispanic Black; Non-Hispanic White versus Asian; and Hispanic versus Asian. In addition, within the high SES stratum, the prevalence of ASD differs at p<0.05 across race/ethnic groups.

## Results

Compared to all 8-year-old children in the study areas, those with ASD were less likely to reside in census block groups classified as poverty areas, and more likely to be male and live in block groups with higher adult educational achievement and a higher MHI (Tables 1 and 2). In addition, among both children with ASD and those in the general study population, there were notable differences in SES by race/ethnicity (Table 2).

The prevalence of ASD increased in a dose-response manner with increasing SES, a pattern seen for all three SES indicators used to define SES categories (Figure 1). When the results were stratified by race/ethnicity, using the % above poverty to define SES categories, significant SES gradients and dose-response increases in ASD prevalence with increasing SES were seen for all strata (Table 3).

**Figure 1:** Prevalence per 1000^1^ of ASD by three SES indicators based on census block group of residence. ^1^Thin bars indicate 95% confidence intervals. Within each SES indicator, both the trend test and χ^2^ tests were significant at p<0.0001. ^2^MHI refers to median household income.

Table 4 presents additional stratified results showing a significant trend toward increasing ASD prevalence with increasing SES: (1) among both boys and girls; (2) regardless of whether there was a pre-existing diagnosis of autistic disorder or an ASD; (3) among children with ASD who did and did not have a history of developmental regression; and (4) regardless of data source (health records only, school records only, and both health and school records). The SES gradient in prevalence, as indicated by the prevalence ratios, was significantly weaker when restricted to children with ASD without a pre-existing autism diagnosis than when restricted to those with a pre-existing diagnosis (p<0.0001, χ^2^ test comparing the SES distribution of cases with and without a pre-existing diagnosis). In addition, when the children with ASD were stratified by the presence or absence of co-occurring cognitive impairment, there was no evidence of an SES gradient in the prevalence of ASD with co-occurring cognitive impairment and a relatively strong gradient in the prevalence of ASD without cognitive impairment (Table 4).

**Table 4:** Stratified Results: ASD and SES^a^ Prevalence Ratios (95% CI^b^), Stratified by Gender, Pre-existing Diagnosis, Co-occurring Intellectual Disability, Developmental Regression, and Data Source.

		ASD Cases		Prevalence Ratios (95% CI)			
		*N* (%)	Living in a Poverty Area^c^ (%)	Low SES	Medium SES	High SES	p-value χ^2^
Total		3680 (100)	16.8	0.70 (0.64, 0.76)	Reference	1.25 (1.16, 1.35)	<0.0001
Gender	Boys	2994 (81.4)	16.3	0.67 (0.60, 0.74)	Reference	1.23 (1.13, 1.34)	<0.0001
	Girls	686 (18.6)	19.0	0.82 (0.67, 1.01)	Reference	1.32 (1.11, 1.57)	<0.0001
Pre-existing ASD Diagnosis	None	1244 (33.8)	19.1	0.78 (0.67, 0.90)	Reference	1.09 (0.94, 1.22)	<0.0001^d^
	ASD (all)	2436 (66.2)	15.7	0.65 (0.58, 0.73)	Reference	1.35 (1.23, 1.48)	<0.0001
	Autistic Disorder	1411 (38.3)	17.8	0.73 (0.63, 0.84)	Reference	1.24 (1.10, 1.40)	<0.0001
	ASD Unspecified	1025 (27.9)	12.8	0.54 (0.45, 0.65)	Reference	1.51 (1.31, 1.73)	<0.0001
Co-occurring Intellectual Disability	Present	1179 (32.0)	22.8	0.86 (0.75, 1.00)	Reference	0.93 (0.81, 1.07)	0.1262
	Absent	1568 (42.6)	14.0	0.52 (0.45, 0.61)	Reference	1.39 (1.25, 1.55)	<0.0001
	Unknown	933 (25.4)	17.6	0.76 (0.64, 0.92)	Reference	1.47 (0.27, 1.71)	<0.0001
Developmental Regression	Present	677 (18.4)	16.4	0.67 (0.54, 0.82)	Reference	1.22 (1.03, 1.45)	<0.0001
	Absent or unknown	3003 (81.6)	16.9	0.70 (0.64, 0.77)	Reference	1.26 (1.16, 1.36)	<0.0001
Source Access^e^	Health & School	1652 (60.9)	15.9	0.65 (0.55, 0.76)	Reference	1.30 (1.14, 1.48)	<0.0001
	Health Only	426 (15.7)	15.1	0.88 (0.67, 1.14)	Reference	1.21 (0.95, 1.54)	<0.0001
	School Only	635 (23.4)	16.0	0.75 (0.64, 0.87)	Reference	1.33 (1.17, 1.52)	<0.0001

a SES indicator is % above poverty level based on United States Census 2000 block group data.

b CI = Confidence Interval.

c Poverty areas include United States Census 2000 block groups in which more than 20% of families with children have incomes below the poverty level [38]. Percent of cases living in poverty is 20.4% in sites accessing only data from healthcare sources.

d In addition to the χ^2^ test of the SES gradient within the stratum of children with no pre-existing ASD diagnosis, a separate χ^2^ test of the difference in the SES gradient for children with and without a pre-existing ASD diagnosis also resulted in a p-value <0.0001.

e Restricted to sites with access to school records (*n* = 2713), including those in Arkansas, Arizona, Colorado, Georgia, Maryland, North Carolina, New Jersey, South Carolina.

## Discussion

This surveillance-based study showed increasing ASD prevalence associated with increasing SES in a dose-response manner, with a stronger SES gradient in ASD prevalence in children with versus without a pre-existing ASD diagnosis. The main results of this study were consistent with the only study larger than this to examine the association between ASD risk and an indicator of SES. That study, published in 2002 by Croen and colleagues, looked at more than 5000 children with autism receiving services coordinated by the California Department of Developmental Services and found a stepwise increase in autism risk with increasing maternal education [13]. Our results were somewhat consistent, but also contrasted somewhat, with Bhasin and Schendel's case-control study based on surveillance data collected in 1996 in Atlanta, Georgia. That study found a positive association between SES and risk of ASD based on ascertainment through health care providers, but not based on ascertainment only from school records [14]. Bhasin and Schendel suggested that this difference by the type of information source might indicate selection bias because in the U.S. access to school-based services is universal whereas access to healthcare is not. In contrast to the Bhasin and Schendel study, our study included a larger number of children with autism identified only from school records (635 vs. 246), was restricted to 8-year-old children (an age at which children with autism are more likely to have been identified, whereas the age range of the Bhasin and Schendel study was 3 through 10 years), and covered the 2002 and 2004 study years (versus 1996, a time when schools were just beginning to use the autism category). Our finding of an SES gradient in autism prevalence regardless of source of information (health vs. school) was not consistent with the hypothesis that the frequency of children with autism identified only through school sources is constant across SES categories. This finding suggests that the observed SES gradient in autism prevalence may not be due entirely to ascertainment bias.

Epidemiologists long have suspected that associations between autism and SES are a result of ascertainment bias, on the assumption that as parental education and wealth increase, the chance that a child with autism will receive an accurate diagnosis also increases [24]. A number of investigators and recent reviews of the epidemiology of autism have concluded that any association observed between autism risk and SES has been due to such bias [26], [27], [30], [31]. The present population-based study of U.S. surveillance data provides some support for this conclusion by showing a stronger SES gradient in prevalence among children with ASD with than without a pre-existing ASD diagnosis. In a previous analysis of ADDM Network data for children identified by the surveillance system as meeting diagnostic criteria for ASD, Mandell and colleagues found non-Hispanic white and Asian children to be more likely than non-Hispanic black and Hispanic children to have a pre-existing ASD diagnosis [39]. In addition to biased ascertainment resulting from those with higher SES having greater access to diagnostic services, it is possible that “diagnostic bias” on the part of clinicians might contribute to ascertainment bias. In a study designed to identify possible diagnostic bias, Cuccaro and colleagues found evidence that clinicians might be more likely to assign autism diagnoses to case vignettes of children with developmental disabilities if the children's backgrounds were described as higher SES rather than lower SES [40]. At the same time, our observation of a significant, if weaker, SES gradient in ASD prevalence when the results are restricted to cases without a pre-existing diagnosis points to the possibility that factors other than ascertainment bias might also contribute to the positive association between ASD prevalence and SES.

A possible reason for the lack of consistency between our findings and those of epidemiologic studies conducted in Denmark [26] and Sweden [27], and which found no association between autism risk and SES, might be that the Scandinavian countries have less socioeconomic diversity and more equitable access to services than the U.S. population. The lack of consistency also could be due to the small number of cases and limited statistical power in the Scandinavian studies, and differences in study designs.

An important advantage of this study was that it was large enough to allow stratified analyses of the association between autism risk and SES among demographic and patient subgroups. It is notable that the SES gradient is observed in all four racial/ethnic strata. Also notable is that, although the overall ASD prevalence was higher among non-Hispanic White and Asian children than among non-Hispanic Black or African-America and Hispanic children, when the results were stratified by SES, we saw that the racial/ethnic differences in prevalence varied by SES (Table 3). The lower prevalence among non-Hispanic Black or African-American and Hispanic children was seen only in the low SES category, and the fact that more non-Hispanic Black or African-American and Hispanic children live in poverty contributed to the lower overall prevalence among these groups.

The only subgroup in which the SES gradient was not observed was the subgroup with co-occurring autism and intellectual disability (Table 4). The lack of an SES association among this subgroup might have been due to counter-associations because intellectual disabilities among children overall are inversely associated with SES [3]. It could also be an indication of ascertainment bias if children with intellectual disabilities are more likely than other children to be evaluated for developmental disorders including autism.

An important limitation of this study was that the ADDM Network surveillance system relies on information for children who have access to diagnostic services for developmental disabilities. We could not rule out the possibility that the quality and quantity of evaluations and information available for case ascertainment might have varied by SES. We looked for evidence of this by examining the number of evaluations per child with ASD recorded in the ADDM Network surveillance system, reasoning that if the higher prevalence of ASD among children of higher SES was due to increased access to diagnostic services, high SES might be associated with a higher number of diagnostic evaluations per child. However, we found no association between the number of evaluations per child and SES. We also examined the mean ages at diagnosis by SES and found that children of high SES received an ASD diagnosis at an average age of 58.0 months, 1.1 month earlier than those of middle SES (p = 0.2838) and 2.7 months earlier than those of low SES (p<0.0272). This modest difference in age at identification may indicate that diagnostic bias contributes to the SES gradient in ASD prevalence in some studies, though not necessarily in the present study which relied on surveillance at the age of eight years and included cases with and without a pre-existing ASD diagnosis.

Another limitation of this study was the reliance on area-level measures of SES that might not have served as accurate proxies for the SES of individuals or specific families or households. Though perhaps not ideal, these measures have been shown to be reasonable proxies for individual-level SES and have the advantage of serving as indicators of the social and economic contexts in which children live but without introducing ecological fallacy [36]. Another limitation of the SES indicators used in this study is that they were based on residential address at the age of eight years rather than at the age of first diagnosis (for children with a pre-existing ASD diagnosis) or other time points, which may have allowed evaluation of whether families of children with ASD migrate to higher SES neighborhoods to improve their access to services, as suggested by Palmer and colleagues [17]. A further limitation of our use of aggregate census data for denominator or comparison group data in this study was that we were unable to perform multivariable analyses to evaluate and control for confounding effects of variables such as parental age and other perinatal risk factors [41].

### Conclusion

If the SES gradient found in this study is due only to ascertainment bias, this would imply that there are significant SES disparities in access to diagnostic and other services for children with autism in communities across the United States. It also would imply that the current estimate of ASD prevalence might be substantially undercounted, with children of low and medium SES being under-identified and underserved relative to those with high SES.

The presence of an attenuated but still statistically significant SES gradient when the analysis was restricted to children with no pre-existing ASD diagnosis suggests the overall SES gradient may not be entirely due to ascertainment bias and points to the possibility that factors associated with socioeconomic advantage might be causally associated with the risk for developing autism. The types of exposures that might merit consideration in future research could include a wide range of factors, from physical or social environmental factors to which children living in more advantaged environments might have higher exposures, to immunological factors (such as that suggested by the “hygiene hypothesis” [42]) or other biological factors (for example, those associated with parental age). It is also possible that the SES association demonstrated in this study was a result of confounding by unknown factors associated with both high SES and susceptibility to ASD, or to effect modification. Further research to identify such factors could lead to advances in our understanding of the etiology and identification of autism and to possible interventions.
